The article "Effect of Nursing Outcome-Oriented Intervention on Airway Management in Elderly Long-Term Bedridden Patients" was retracted in 2023. Reasons: signs of a paper mill; compromised peer review; unreliable results or conclusions.

# Effect of Nursing Outcome-Oriented Intervention on Airway Management in Elderly Long-Term Bedridden Patients

**DOI:** 10.1155/2022/9557330

**Published:** 2022-10-11

**Authors:** Weiwei Ding, Fei Luo, Pingping Lin, Yu Tang, Ying Liu

**Affiliations:** ^1^Department of Neurosurgery, Yantai Affiliated Hospital of Binzhou Medical University, Yantai, Shandong 264100, China; ^2^Department of Gastrointestinal Surgery, Yantai Affiliated Hospital of Binzhou Medical University, Yantai, Shandong 264100, China; ^3^Department of Obstetrics, Yantai Affiliated Hospital of Binzhou Medical University, Yantai, Shandong 264100, China; ^4^College of Basic Medicine, Binzhou Medical University, Yantai, Shandong 264000, China

## Abstract

**Objective:**

This study intended to explore the nursing outcome-oriented intervention's effect on airway management in elderly long-term bedridden patients.

**Methods:**

A total of 120 cases of elderly long-term bedridden patients admitted to our hospital from May 2018 to June 2020 were enrolled and randomly divided into the observation group (*n* = 60) and control group (*n* = 60). The control group received the routine nursing intervention, while the observation group received the nursing outcome-oriented intervention. Forced expiratory volume (FEV1), forced vital capacity (FVC), and maximal voluntary ventilation (MVV) in the first second were compared between the two groups before and after the intervention. The pulmonary infection of the two groups was observed. Total protein, hemoglobin, albumin, and cholesterol levels were compared between the two groups. Hamilton Anxiety Scale (HAMA) and Hamilton Depression Scale (HAMD) were used to evaluate the two groups' psychological status before and after the intervention. The Generic Quality of Life Inventory-74 (GQOLI-74) assessed the two groups' quality of life.

**Results:**

After the intervention, the levels of FEV1, FVC, and MVV; total protein, hemoglobin, albumin, and cholesterol; and scores of physical function, psychological function, social function, and material life function in the observation group were higher than those in the control group. Pulmonary infection, secondary infection, the infection rate is more than 3%, HAMA, and HAMD scores, and the incidence of pressure ulcers, aspiration, constipation, and the falling bed was lower than those in the control group, with statistical significance (all *P* < 0.05).

**Conclusion:**

Nursing outcome-oriented intervention can effectively improve lung function, pulmonary infection, nutritional status, negative mood, and quality of life of long-term bedridden elderly patients.

## 1. Introduction

Older adults often need to stay in bed for a long time because of a weak physique or chronic diseases, but the long-term bedridden states can cause complications such as pulmonary infection and pressure sores, which seriously affect the quality of life of patients. Without professional nursing care, these elderly patients generally develop hypostatic pneumonia after long-term bed rest; moreover, reduced or lost function of humidification and heating of upper respiratory mucosa of elderly patients can result in difficult expectoration of astringent or sticky sputum, swallowing reflex, and hypesthesia of laryngeal mucosa, causing aspiration. The establishment of an artificial airway is designed to improve the respiratory function of patients, alleviate respiratory disorders, and assist in the clearance of respiratory secretions. Improper nursing of the artificial airway will significantly reduce its use and therapeutic effect, increase the risk of related adverse reactions, and even endanger patients' lives. Therefore, effective airway management based on the physical condition and psychological characteristics of the elderly is of great importance. Although conventional nursing intervention can help patients reduce stress reactions to a certain extent, it follows the established model for the patient taking care of them. The end of nursing means that the patient ends after the care intervention. It can measure whether the nursing method is effective and help the nursing staff make clinical decisions; that is, nursing staff can improve and implement the existing and potential patient problems during the treatment process. Nursing outcome-oriented nursing intervention differs from conventional nursing based on the patient's physical and psychological states. In nursing outcome-oriented nursing intervention, the nursing outcome should be selected first, followed by nursing with the outcome as the target, improving nursing efficiency and patients' prognosis and quality of life [1–4].

The article "Effect of Nursing Outcome-Oriented Intervention on Airway Management in Elderly Long-Term Bedridden Patients" was retracted in 2023. Reasons: signs of a paper mill; compromised peer review; unreliable results or conclusions.

This study was aimed at investigating the effect of the nursing outcome-oriented intervention on airway management in elderly patients with long-term bedridden conditions.

## 2. Material and Methods

### 2.1. General Data

One hundred twenty elderly long-term bedridden patients admitted to our hospital from May 2018 to June 2020 were recruited and randomly divided into the observation and control groups, with 60 cases in each group. In the observation group, there were 38 males and 22 females. The age ranged from 65 to 88 years, with an average age of 75.53 ± 5.94. The bed stay ranged from 1 to 16 months, with an average of 9.85 ± 2.43 months. The following are the primary disease types: cerebral hemorrhage in 24 cases, cerebral infarction in 32 cases, and lower limb fracture in 4 cases. In the control group, there were 42 males and 18 females. The age was from 65 to 88 years, with an average age of 74.78 ± 4.39 years. The average bed stay ranged from 1 to 15 months, with an average of 9.17 ± 3.14 months. The following are the primary disease types: cerebral hemorrhage in 27 cases, cerebral infarction in 28 cases, and lower limb fracture in 5 cases. The general data of the two groups were comparable (all *P* > 0.05). This study was approved by the hospital ethics committee.

### 2.2. Inclusion Criteria

The following are the inclusion criteria: (1) clear clinical diagnosis, (2) stay in bed ≥ 1 month, (3) complete clinical data, and (4) voluntary participation.

### 2.3. Exclusion Criteria

The following are the exclusion criteria: (1) Patients with mental diseases or consciousness disorders; (2) patients with severe deterioration of the primary disease; (3) patients with severe immune dysfunction; (4) patients with congenital heart disease, liver and kidney insufficiency, coagulation dysfunction, and malignant tumor diseases; (5) patients with severe respiratory tract infection and pressure ulcers at the time of admission; and (6) patients with insufficient nursing compliance.

### 2.4. Grouping

#### 2.4.1. Control Group

The control group was given routine nursing. After admission, patients and their families received conventional health education. Patients were told the precautions, including diet, during bed rest treatment, and given routine airway management, routine massage nursing, and routine psychological counseling. During the stay in bed, nurses observed patients' airway status to observe whether there was a lung infection, patted patients' back to help maintain normal respiratory function, and instructed the family members to carry out relevant training. The patient's symptoms were closely watched, and discomfort should be reported to the doctor in time.

#### 2.4.2. Observation Group

The observation group received the nursing outcome-oriented intervention, and the nursing goals were set according to nursing outcomes. The evaluation indexes of nursing outcomes include physical health, functional health, psychological and social health, perceived health, knowledge and behavior, family health, and community health. In this study, they can be summarized into three areas: (1) improving patients' bad moods; (2) improving patients' airway function—(a) body posture management, (b) cough and expectoration, (c) airway humidification, and (d) respiratory function training; and (3) improving the quality of life of patients—(a) nutrition support, (b) prevention of falling into bed, (c) prevention of venous thrombosis, and (d) prevention of constipation.

The article "Effect of Nursing Outcome-Oriented Intervention on Airway Management in Elderly Long-Term Bedridden Patients" was retracted in 2023. Reasons: signs of a paper mill; compromised peer review; unreliable results or conclusions.

### 2.5. Observation Targets

The following are the observation targets:

1. Pulmonary function indices: forced expiratory volume in the first second (FEV1), forced vital capacity (FVC), and maximal voluntary ventilation (MVV) were compared between the two groups before and after the intervention.
2. Whether the patient has a pulmonary infection
3. Nutritional state: before and after the intervention, the fasting venous blood was taken from patients in the morning to detect the total protein, hemoglobin, albumin, and cholesterol levels in both groups.
4. Mental state: Hamilton Anxiety Scale (HAMA) [5] and Hamilton Depression Scale (HAMD) [6] were used to evaluate the two groups' psychological status before and after the intervention. HAMA includes 14 entries and can be graded as five levels: no anxiety (0~7 points), suspected anxiety (8~14 points), anxiety (15~21 points), moderate anxiety (22~29 points), and severe anxiety (≥30 points). HAMD includes 24 entries and can be graded as three levels: no depression (0~8 points), mild to moderate depression (21~35 points), and severe depression (≥36 points).
5. Whether the patient has any adverse reactions
6. Quality of life: Generic Quality of Life Inventory-74 (GQOLI-74) [7] was used to evaluate the quality of life of the two groups before and after the intervention, consisting of 64 items in 4 dimensions. The maximum score for each dimension is 80, and the higher the score, the better the quality of life.

### 2.6. Statistical Approaches

All data in this study were input into an Excel table by two people without communication and analyzed by statistical software SPSS24.0. Measurement data were expressed as the mean ± SD and tested by a *t*-test when they were in line with normal distribution and had equal variance. Counting data were described by *n* and %, and the chi-square test was used to compare groups. All tests were two-sided, and *P* < 0.05 was considered statistically significant.

## 3. Results

### 3.1. Comparison of Lung Function between the Two Groups

Before the intervention, no significant differences between the two groups were seen in FEV1, FVC, and MVV levels (all *P* > 0.05). After the intervention, the levels of FEV1, FVC, and MVV in both groups were increased, and the improvement degree of each indicator in the observation group was greater than that in the control group (*P* > 0.05) (Table 1).

### 3.2. Comparison of Pulmonary Infection between the Two Groups

The pulmonary infection, secondary infection, and infection rate of more than 3% in the observation group were significantly lower than in the control group (all *P* < 0.05, Table 2).

The article "Effect of Nursing Outcome-Oriented Intervention on Airway Management in Elderly Long-Term Bedridden Patients" was retracted in 2023. Reasons: signs of a paper mill; compromised peer review; unreliable results or conclusions.

### 3.3. Comparison of Nutritional Status between the Two Groups

Before the intervention, no significant differences between the two groups were observed in total protein, hemoglobin, albumin, and cholesterol levels (all *P* > 0.05). After the intervention, the levels of total protein, hemoglobin, and albumin in both groups increased, and the levels of total protein, hemoglobin, albumin, and cholesterol in the observation group were significantly higher than those in the control group (all *P* < 0.05) (Table 3).

### 3.4. Comparison of Psychological States between the Two Groups

Before the intervention, the two groups had no significant differences in HAMA and HAMD scores (*P* > 0.05). After the intervention, HAMA and HAMD scores were decreased in both groups, and the observation group was lower than the control group, with statistical significance (both *P* < 0.05) (Table 4).

### 3.5. Comparison of Adverse Events between the Two Groups

The incidence of pressure sores, aspiration, constipation, and falling bed in the observation group was significantly lower than in the control group, and the differences were statistically (all *P* < 0.05, Table 5).

### 3.6. Comparison of Quality of Life between the Two Groups

Before the intervention, no significant differences were seen in scores of physical, psychological, social, and material life function scores between the two groups (all *P* > 0.05). After the intervention, the scores of psychological function, social function, and material life function increased in both groups, and the scores of these indices of the observation group were higher than those of the control group, with statistical significance (all *P* < 0.05) (Table 6).

## 4. Discussion

With the progress of population aging, the demand for hospital treatment and nursing of elderly patients is rising gradually. The common diseases of elderly patients, such as cardiovascular and cerebrovascular diseases, chronic diseases, and fractures, need long-term bed treatment, which can cause various complications [8–10]. For elderly patients with poor physical reserve ability, even a short time in bed may adversely affect the body. The circulatory, respiratory, digestive, skin, and other aspects of elderly long-term bedridden patients can vary. Moreover, patients who stay in bed for a long time are unable to carry out necessary social communication, and long-term loneliness can affect the psychological state of patients, resulting in anxiety and depression over time, further affecting the prognosis of patients. Swallowing reflexes and hypesthesia of laryngeal mucosa may also lead to aspiration and lung infection, so attention should be paid to airway management in long-term bedridden elderly patients [11, 12]. In this study, the observation group received nursing outcome-oriented nursing, while the control group received routine nursing. The results showed that the levels of FEV1, FVC, and MVV in the observation group were higher than those in the control group. FEV1 is the volume of air exhaled in the first second of exhalation. FVC is the maximum volume of air a person can exhale, and FEV1 and FVC are often used as pulmonary function indicators in clinical practice [13, 14]. The levels of FEV1 and FVC in ordinary people are about 83%. Too high or too low levels indicate abnormalities. MVV is the maximum volume, and its value is related to factors such as airway patency and respiratory muscle strength [15]. In the present study, the improvement degree of FEV1, FVC, and MVV levels in the observation group was more remarkable than that in the control group, proving that the effect of nursing outcome-oriented nursing on lung function improvement of the long-term bedridden elderly patients is better than that of conventional nursing. Nursing outcome-oriented nursing outcomes were summarized into three areas: improving patients' negative mood, improving patients' airway function, and improving patients' quality of life. Then, targeted nursing was carried out based on the nursing outcomes. The improvement of lung function in the observation group may be related to respiratory function training in improving patients' airway function. In this study, the pulmonary infection, secondary infection, and ≥3 infection rate in the observation group were all lower than those in the control group, indicating that nursing outcome-oriented nursing intervention had a better effect than conventional nursing in reducing the pulmonary infection rate in the elderly long-term bedridden patients. In the nursing intervention guided by nursing results, posture management, cough expectoration, and airway humidification can effectively promote patients to cough up phlegm. Difficulty in expectoration can easily lead to pulmonary infection, so promoting expectoration is conducive to reducing the incidence of pulmonary infection.

The article "Effect of Nursing Outcome-Oriented Intervention on Airway Management in Elderly Long-Term Bedridden Patients" was retracted in 2023. Reasons: signs of a paper mill; compromised peer review; unreliable results or conclusions.

Comparisons of the nutritional status after intervention showed that the levels of nutritional indicators such as total protein, hemoglobin, albumin, and cholesterol in the observation group were higher than those in the control group, indicating that nursing outcome-oriented nursing intervention can effectively improve the nutritional status of patients. Chronic bedridden patients may be accompanied by dysphagia, leading to malnutrition and insufficient nutritional intake, affecting patient outcomes. Therefore, proper nutritional support is beneficial to reducing complications and promoting patients' recovery. Improving patients' quality of life in nursing outcome-oriented nursing intervention includes nutritional support for elderly patients, and in vitro nutritional support for patients with eating difficulties can ensure adequate nutrition during hospitalization. In this study, HAMA and HAMD scores of the observation group were lower than those of the control group after the intervention, indicating that nursing outcome-oriented nursing intervention had a better effect on improving patients' bad moods than conventional nursing. Previous studies have shown that a bad mood can affect the recovery of patients [16–18]. In the present study, a nursing outcome-oriented nursing intervention is aimed at improving patients' adverse emotional outcomes. The downbeat mood of the long-term bedridden elderly patients was effectively improved by encouraging them with words and creating a good atmosphere in the wards. Previous studies have demonstrated that long-term bed rest can cause multiple complications, such as pressure sores and constipation [19, 20]. Elderly patients are also prone to falling beds. Elderly patients have poor physical function, and falling into bed can lead to severe consequences. In the present study, the incidence of pressure sores, aspiration, constipation, and falling bed in the observation group was lower than that in the control group, indicating that nursing outcome-oriented nursing intervention can effectively reduce the incidence of adverse events in long-term bedridden elderly patients. The nursing outcome-oriented nursing intervention is aimed at “improving patients' quality of life.” Based on the characteristics of long-term bed rest, nursing interventions targeted to prevent falling bed, venous thrombosis, and constipation were given. In addition, airway management was also conducive to preventing aspiration, effectively reducing adverse events. After the intervention, the scores of physical, psychological, social, and material life functions of the observation group were higher than those of the control group, indicating that nursing outcome-oriented nursing intervention can effectively improve patients' quality of life. The part of “improving patients' quality of life” in the nursing outcome-oriented nursing intervention, nutritional support, and prevention of adverse events was provided to patients, effectively improving the nutritional status of patients and reducing the occurrence of adverse events.

In conclusion, nursing outcome-oriented intervention can effectively improve the lung function and nutritional status of long-term bedridden elderly patients, relieve their negative mood, improve their quality of life, and reduce the occurrence of adverse events such as infection and complications, showing clinical application value.

The article "Effect of Nursing Outcome-Oriented Intervention on Airway Management in Elderly Long-Term Bedridden Patients" was retracted in 2023. Reasons: signs of a paper mill; compromised peer review; unreliable results or conclusions.

## Figures and Tables

**Table 1:** Comparison of lung function between the two groups ($\bar{x}\pm s$).

Group	FEV1 (%)		FVC (%)		MVV (L/min)	
	Before intervention	After intervention	Before intervention	After intervention	Before intervention	After intervention
Observation group (*n* = 60)	37.34 ± 4.05	48.78 ± 4.43^a^	62.01 ± 5.31	68.77 ± 5.98^a^	78.39 ± 4.36	85.07 ± 6.45^a^
Control group (𝑛 =60)	37.27 ± 3.63	41.99 ± 3.51^a^	60.53 ± 4.53	63.18 ± 5.21^a^	78.31 ± 5.27	79.63 ± 6.17^a^
*t* value	0.107	9.298	1.646	5.450	0.096	4.719
*P* value	0.915	<0.001	0.102	<0.001	0.924	<0.001

Compared with the same group before the intervention, ^a^*P* < 0.05.

**Table 2:** Comparison of pulmonary infection between the two groups [cases (%)].

Group	Pulmonary infection	Secondary infection	More than 3%	Ventilator use
Observation group (*n* = 60)	29 (48.33)	20 (33.33)	14 (23.33)	3 (5.00)
Control group (*n* = 60)	50 (83.33)	42 (70.00)	36 (60.00)	7 (11.67)
*χ* ^2^ value	16.338	16.151	16.594	1.745
*P* value	<0.001	<0.001	<0.001	0.186

**Table 3:** Comparison of nutritional status between the two groups ($\bar{x}\pm s$).

Group	Total protein (g/l)		Hemoglobin (g/l)		Albumin (g/l)		Cholesterol (mmol/l)	
	Before intervention	After intervention	Before intervention	After intervention	Before intervention	After intervention	Before intervention	After intervention
Observation group (*n* = 60)	51.95 ± 7.22	58.52 ± 5.25^a^	103.23 ± 16.51	109.55 ± 9.04^a^	178.34 ± 40.91	213.22 ± 58.52^a^	3.12 ± 0.98	4.07 ± 0.87^a^
Control group (*n* = 60)	53.29 ± 5.26	55.51 ± 5.44^a^	103.44 ± 11.34	104.80 ± 13.63^a^	176.12 ± 55.38	179.42 ± 48.34^a^	3.35 ± 0.86	3.34 ± 1.17
*t* value	1.164	3.076	0.083	2.251	0.250	3.449	1.396	3.849
*P* value	0.247	0.003	0.934	0.027	0.803	0.001	0.165	<0.001

Compared with the same group before the intervention, ^a^*P* < 0.05.

**Table 4:** Comparison of psychological states between the two groups ($\bar{x}\pm s$).

Group	HAMA score		HAMD score	
	Before intervention	After intervention	Before intervention	After intervention
Observation group (*n* = 60)	18.52 ± 1.90	11.53 ± 1.02^a^	16.75 ± 1.60	9.70 ± 0.96^a^
Control group (*n* = 60)	18.23 ± 1.76	16.75 ± 1.63^a^	17.15 ± 1.45	14.42 ± 1.00^a^
*t* value	0.847	21.013	1.435	26.378
*P* value	0.398	<0.001	0.154	<0.001

Compared with the same group before the intervention, ^a^*P* < 0.05.

**Table 5:** Comparison of adverse events between the two groups [cases (%)].

Group	Pressure sores	Aspiration	Constipation	Falling bed
Observation group (*n* = 60)	6 (10.00)	10 (16.67)	17 (28.33)	4 (6.67)
Control group (*n* = 60)	32 (53.33)	42 (70.00)	45 (75.00)	19 (31.67)
*χ* ^2^ value	26.033	34.751	26.162	12.102
*P* value	<0.001	<0.001	<0.001	<0.001

The article "Effect of Nursing Outcome-Oriented Intervention on Airway Management in Elderly Long-Term Bedridden Patients" was retracted in 2023. Reasons: signs of a paper mill; compromised peer review; unreliable results or conclusions.

**Table 6:** Comparison of quality of life between the two groups (*x* ± *s*, points).

Group	Physical function		Mental function		Social function		The function of material life	
	Before intervention	After intervention	Before intervention	After intervention	Before intervention	After intervention	Before intervention	After intervention
Observation group (*n* = 60)	45.70 ± 4.39	51.27 ± 7.62^a^	46.07 ± 4.72	70.38 ± 6.71^a^	45.90 ± 4.81	65.83 ± 5.70^a^	49.52 ± 4.85	68.25 ± 6.09^a^
Control group (*n* = 60)	46.47 ± 5.13	47.42 ± 5.81	47.62 ± 4.61	54.97 ± 6.88^a^	46.52 ± 4.51	57.80 ± 5.99^a^	51.12 ± 6.06	62.60 ± 6.47^a^
*t* value	0.879	3.112	1.820	12.423	0.724	7.527	1.597	4.926
*P* value	0.381	0.002	0.071	<0.001	0.470	<0.001	0.113	<0.001

Compared with the same group before the intervention, ^a^*P* < 0.05.

## Data Availability

The labeled dataset used to support the findings of this study is available from the corresponding author upon request.
